# Impact of the COVID-19 Pandemic on Physical Therapy Clinical Practice in Egypt: A Cross-Sectional Study

**DOI:** 10.7759/cureus.73507

**Published:** 2024-11-12

**Authors:** Hosny Elkhawaga, Abdallah M Kamel, Mohamed Badr, Abdallah Gamiel, Ahmed A Basheer

**Affiliations:** 1 Faculty of Physical Therapy, Cairo University, Giza, EGY; 2 Medical Research Group of Egypt, Negida Academy, Arlington, USA; 3 Department of Physical Therapy for Musculoskeletal Disorders and Its Surgeries, Faculty of Physical Therapy, Cairo University, Giza, EGY; 4 Department of Physical Therapy for Neuromuscular Disorders and Its Surgery, Faculty of Physical Therapy, Al Hayah University in Cairo, Cairo, EGY; 5 Department of Physical Therapy for Musculoskeletal Disorders and Its Surgery, Faculty of Physical Therapy, Modern University for Technology and Information (MTI) University, Cairo, EGY; 6 Department of Physical Therapy for Musculoskeletal Disorders, Faculty of Physical Therapy, Beni Suef University, Beni Suef, EGY

**Keywords:** clinical practice, coronavirus disease 2019 (covid-19), covid-19, covid-19 pandemic, egypt, physical therapy specialty, physiotherapy management, physiotherapy rehabilitation, sars-cov-2 (severe acute respiratory syndrome coronavirus 2)

## Abstract

Background

The coronavirus disease 2019 (COVID-19) was an expanding pandemic caused by a new strain of the coronavirus family known as severe acute respiratory syndrome coronavirus 2 (SARS-CoV-2). No previous studies have examined the impact of COVID-19 pandemic on physical therapy practice in Egypt.

Objectives

This study aimed to assess the impact of COVID-19 pandemic on physical therapy clinical practice in Egypt five months after the pandemic declaration. The study investigated how Egyptian physical therapists interacted during the pandemic and the effect of the pandemic on precautionary measures. Additionally, this study assessed the knowledge of physical therapists about COVID-19.

Methods

A cross-sectional study with a convenient sample was conducted in Egypt through an online structured questionnaire. Data were collected between August 28, 2020, and October 10, 2020.

Results

A total of 409 physical therapists from 23 Egyptian governorates completed the survey. At some point during the COVID-19 pandemic, 249 (60.9%) physical therapists left their work. Only 131 (32%) visited patients' homes. The majority of respondents, 330 (80.7%), reported that they were afraid to catch any infection from patients during assessment and treatment. Moreover, 330 (80.7%) reported feeling anxious about the COVID-19 pandemic, and 220 (53.8%) reported that their mental health and well-being were not okay. The majority of the participants committed to precautionary measures of physical therapists during the COVID-19 pandemic. The mean knowledge score was 18.29±1.99 out of 23.

Conclusions

The COVID-19 pandemic affected physical therapy clinical practice in Egypt. It had a psychological impact on Egyptian physical therapists. Egyptian physical therapists committed to precautionary measures against COVID-19 and demonstrated a very good knowledge about COVID-19. Physical therapists should be aware of precautionary measures against infectious diseases, which help can prevent the spread of disease if any new pandemic occurs.

## Introduction

The coronavirus disease 2019 (COVID-19) was an expanding pandemic caused by a new strain of the coronavirus family known as severe acute respiratory syndrome coronavirus 2 (SARS-CoV-2) [1]. Coronaviruses family causes illnesses that may be mild, such as the common cold, or severe, such as severe acute respiratory syndrome (SARS-CoV) and Middle East Respiratory Syndrome (MERS-CoV), which emerged in 2003 and 2012, respectively [2]. In December 2019, COVID-19 began in Wuhan city in China and then spread all over the world. COVID-19 kept spreading until the World Health Organization (WHO) declared it a pandemic on March 11, 2020. Five months after the pandemic declaration, by August 11, 2020, there were approximately 20.5 million cases globally, including around 744,000 deaths due to COVID-19. In Egypt, there were around 96,000 cases and more than 5,000 deaths. Egypt reported its peak of cases (1,774) and deaths (97) on June 19 and June 15, respectively. Then, the numbers began to decrease to reach 168 cases and 24 deaths on August 11, 2020 [3].

COVID-19 is transmitted from an affected person to a healthy one by close contact via respiratory droplets during coughing or sneezing. Older adults and patients with chronic illnesses are at increased risk of infection and serious complications [4,5]. Regarding the clinical symptoms of COVID-19, fever is the most common one. Symptoms also include cough, shortness of breath, malaise, and fatigue [2]. In severe cases, COVID-19 causes pneumonia similar to the fatal one caused by SARS-CoV and MERS-CoV [6]. At the time of data collection for this study, no approved vaccination or treatment for COVID-19 was available. Therefore, following the precautionary measures was the primary intervention to limit the spread of COVID-19 either in the community or health care setting [7]. Regarding the clinical practice of outpatient physical therapists, the American Physical Therapy Association (APTA) recommends wearing a face mask, using gloves in case of patient contact procedures, disinfecting equipment between each patient, and washing hands after, before, and between each session. Screening the patient's temperature before each session is also necessary [8].

In addition to changing the psychological and mental status of the general population and medical staff, COVID-19 affected the clinical practice of different medical specialties worldwide [9-11]. Inadequate knowledge and improper infection control measures among healthcare workers can lead to the spread of disease, as occurred with MERS-CoV [12]. Previous studies indicate that the Egyptian population and healthcare workers generally have good knowledge about COVID-19 [13,14]. To the best of our knowledge, no previous studies have examined the impact of COVID-19 pandemic on physical therapy practice in Egypt. Therefore, this study aimed to assess the impact of COVID-19 pandemic on physical therapy clinical practice in Egypt five months after the pandemic declaration. The study investigated how Egyptian physical therapists interacted during the pandemic and the effect of the pandemic on precautionary measures. Additionally, this study assessed the knowledge of physical therapists about COVID-19.

## Materials and methods

Study design and ethics

A cross-sectional study with a convenient sample was conducted in Egypt through an online structured questionnaire. Data were collected between August 28, 2020, and October 10, 2020. This study was approved by the Ethical Committee of the Faculty of Physical Therapy, Cairo University, Cairo, Egypt (No: P.T.REC\012\004186). The online questionnaire included an informed consent, which participants had to read and accept to participate before answering the questions.

Study population

Both male and female physical therapists working in any clinical practice setting in any Governorate in Egypt were eligible for the study. Physical therapy students and physical therapists who were not practicing physical therapy, such as academics and managers, were excluded.

Instruments and data collection

A structured self-administered questionnaire was designed to fulfil the objectives of the study. The questionnaire was developed using Google Forms and distributed online via social media applications. This questionnaire consisted of the following four sections:

Demographic characteristics of respondents: This section included gender, age, governorate of work, area of work, level of education, years of experience, scope of practice, and workplace.

Interaction of physical therapists during the COVID-19 pandemic: Five questions were included in this part. These questions were about work leaving, home visits, fear of infection, anxiety, and mental health.

Precautionary measures of physical therapists during the COVID-19 pandemic: Questions in this section were designed based on Considerations for Outpatient Physical Therapy Clinics During the COVID-19 Public Health Crisis produced by the APTA [8]. This section included eight questions about committing patients to wear face masks, committing patients to sterilizing their hands, screening patients' temperature, wearing face masks, wearing hand gloves, washing hands, and cleaning and sterilizing assessment and treatment area.

Knowledge of physical therapists about COVID-19: Questions in this section were adapted from the survey questions used in a previous study, which assessed knowledge regarding COVID-19 [13]. This part included 23 questions on COVID-19 transmission, symptoms, and prevention. The correct answer was scored 1 point, the maximum score was 23, and the minimum was 0.

The questionnaire used in this study is included in the Appendix.

Sample size calculation

Sample size was calculated using Epi Info™ software. Under a 95% confidence level, 0.05 margin of error, and assumed 50% of expected frequency, a sample of 384 participants was considered as a minimum sample.

Statistical analysis

Data analyses were conducted using SPSS Version 25 (IBM Corp., Armonk, NY, USA). Descriptive statistics was used to summarize data on the demographics of survey respondents, interaction during the COVID-19 pandemic, precautionary measures during the COVID-19 pandemic, and knowledge about COVID-19. Data were presented as frequencies (n) and percentages (%) for all categorical variables and means ± standard deviation for numerical variables.

## Results

Study participants

A total of 409 physical therapists from 23 Egyptian governorates completed the survey. There were 162 (39.6%) males and 247 (60.4%) females. In terms of age, 222 (54.3%) were <30 years of age, 167 (40.8%) were 30-39 years of age, and 20 (4.9%) were ≥40 years of age. The majority of the respondents (50.4 %) were bachelor's degree holders, 21% and 5.1% completed their master of science (MSc) degree and doctor of philosophy (PhD) degree, respectively. Moreover, 371 (90.7%) of the participants worked in an urban area, whereas only 38 (17.7 %) stated working in a rural area. The mean years of experience of the participants was 7.63 ± 5.59 years. The most commonly practiced specialty was orthopedics 324 (79.2%). The majority of the respondents worked in Ministry of Health and Population hospitals 265 (64.8%) and private centers 267 (65.3%). Demographics of survey respondents are shown in Table 1.

**Table 1:** Demographics of survey respondents (n=409) *Multiple responses were allowed. SD, standard deviation; DPT, doctor of physical therapy; MSc, master of science; PhD, doctor of philosophy; MOHP, Ministry of Health and Population

	N	%
Gender		
Male	162	39.6
Female	247	60.4
Age (years)		
<30	222	54.3
30-39	167	40.8
≥40	20	4.9
Mean ± SD	29.66 ± 5.4	
Governorate of work		
Cairo	112	27.4
Dakahlia	42	10.3
Giza	41	10
Alexandria	28	6.8
Gharbia	27	6.6
Kafr El Sheikh	22	5.4
Others	137	33.5
Area of work		
Urban	371	90.7
Rural	38	9.3
Level of education		
Intern	43	10.5
Bachelor's degree	206	50.4
DPT degree	53	13
MSc degree	86	21
PhD degree	21	5.1
Years of experience		
≤5	178	43.5
6-10	129	31.5
11-15	66	16.1
>15	36	8.8
Mean ± SD	7.63 ± 5.59	
Scope of practice^*^		
Orthopedics	324	79.2
Neurology	205	50.1
Pediatrics	147	35.9
Sports	146	35.7
Geriatrics	43	10.5
Cardiovascular and pulmonary	34	8.3
Women's health	34	8.3
Wound management	13	3.2
Others	105	25.7
Workplace^*^		
MOHP hospitals	265	64.8
University hospitals	44	10.8
Private centers	267	65.3
Others	74	18.1

Interaction of physical therapists during the COVID-19 pandemic

Overall, 249 (60.9%) physical therapists left their work at some point during the COVID-19 pandemic. Only 131 (32%) visited patients' homes. The majority of respondents, 330 (80.7%), reported that they were afraid to catch an infection from patients during assessment and treatment. Moreover, 330 (80.7%) reported feeling anxious about the COVID-19 pandemic, and 220 (53.8%) reported that their mental health and well-being were not okay. The interaction of physical therapists during the COVID-19 pandemic is shown in Table 2.

**Table 2:** Interaction of physical therapists during the COVID-19 pandemic (n=409)

	Yes		No	
	N	%	N	%
Did you leave your work as a physical therapist at any period during the COVID-19 pandemic?	249	60.9	160	39.1
Do you visit your patient's home "home physiotherapy," if requested?	131	32	278	68
Are you afraid to catch any infection from patients during assessment and treatment?	330	80.7	79	19.3
Do you feel anxiety about the COVID-19 pandemic?	330	80.7	79	19.3
Do you feel that your mental health and well-being are not okay?	220	53.8	189	46.2

Precautionary measures of physical therapists during the COVID-19 pandemic

Generally speaking, the majority of the participants committed to precautionary measures of physical therapists during the COVID-19 pandemic, as shown in Table 3.

**Table 3:** Precautionary measures of physical therapists during the COVID-19 pandemic (n=409)

	Yes		No	
	N	%	N	%
Committing patients to wear face masks	375	91.7	34	8.3
Committing patients to sterilize their hands before assessment and treatment	301	73.6	108	26.4
Screening patient temperature	167	40.8	242	59.2
Wearing face mask	385	94.1	24	5.9
Wearing hand gloves	337	82.4	72	17.6
Washing hands before and after every patient	367	89.7	42	10.3
Cleaning and sterilizing assessment and treatment area including plinths, tools, and equipment before and after every patient	361	88.3	48	11.7
Modifying techniques to keep social distance	298	72.9	111	27.1

Knowledge of physical therapists about COVID-19

The total knowledge score ranged from 10 to 22, with a mean of 18.29 ± 1.99. Results of the knowledge assessment of physical therapists regarding COVID-19 transmission, symptoms, and preventive measures are shown in Table 4.

**Table 4:** Knowledge assessment of physical therapists about COVID-19 (n=409) *Correct answer

	Yes		No	
	N	%	N	%
COVID-19 spreads by				
1. Droplets of an affected person (with cough or expiration)	393^*^	96.1	16	3.9
2. Surfaces touched by an affected person	332^*^	81.2	77	18.8
3. Touching coins and banknotes	245	59.9	164^*^	40.1
4. Dealing with pets	44	10.8	365^*^	89.2
5. Stool (e.g., in public toilets)	76	18.6	333^*^	81.4
6. Goods imported from China	43	10.5	366^*^	89.5
7. The disease could be transmitted from an asymptomatic person	270^*^	66	139	34
Common symptoms include				
8. Fever	392^*^	95.8	17	4.2
9. Dry cough	354^*^	86.6	55	13.4
10. Body aches	222^*^	54.3	187	45.7
11. Difficulty in breathing	346^*^	84.6	63	15.4
12. Vomiting	116	28.4	293^*^	71.6
13. The virus may be more dangerous for the elderly	366^*^	89.5	43	10.5
14. The virus may be more dangerous in patients with chronic diseases	376^*^	91.9	33	8.1
Measures to prevent the spread of the disease include				
15. Proper hand wash	379^*^	92.7	30	7.3
16. Maintaining an appropriate distance between yourself and anyone with symptoms	388^*^	94.9	21	5.1
17. Avoiding touching eyes, nose, and mouth	373^*^	91.2	36	8.8
18. Putting on facemasks in public places	386	94.4	23^*^	5.6
19. Taking antibiotics	31	7.6	378^*^	92.4
20. Eating garlic	87	21.3	322^*^	78.7
21. An effective vaccine against the virus is currently available	20	4.9	389^*^	95.1
22. An effective treatment against the virus is currently available	77	18.8	332^*^	81.2
23. Antibiotics can treat the disease	85	20.8	324^*^	79.2
Total score				
Mean ± SD	18.29 ± 1.99			
Median (IQR)	19 (17-20)			
Min–max	(10-22)			

## Discussion

Our study showed that COVID-19 pandemic affected physical therapy clinical practice in Egypt. Egyptian physical therapists interacted during the pandemic and committed to precautionary measures against COVID-19. Additionally, they demonstrated a very good knowledge about COVID-19.

Due to the high outbreak of COVID-19, this survey showed that physical therapists were panicking about the pandemic. Around 61% left their work as physical therapists at a period during the pandemic, and 68% refused to visit their patients at home. Furthermore, around 81% of them were afraid to catch any infection from patients during assessment and treatment, and the same percentage was anxious. Moreover, 53.8% reported that their mental health and well-being were not okay. The psychological impact of COVID-19 outbreak on healthcare workers has been reported in the literature. Previous studies reported an adverse psychological impact including anxiety and depression on healthcare workers [15,16]. Additionally, Elsayed et al. demonstrated that the pandemic made Saudi physical therapists suffer from notable psychological stress [17].

The study showed that the pandemic has significantly affected the stringent precautionary measures taken by the most of participating physical therapists during the assessment and treatment sessions [8]. Most of them ordered their patients to wear face masks and sterilize their hands before assessment and treatment. Almost 41% of them screened their patients’ temperatures. Additionally, most physical therapists committed to wearing face masks and hand gloves and washing hands before and after every patient, as well as cleaning and sterilizing the assessment and treatment area including plinths, tools, and equipment before and after every patient. Furthermore, around 73% of them modified the treatment techniques to keep social distancing, which reflects the severe fear of catching infection from the patients.

Adequate knowledge about COVID-19 could help prevent the spread of the disease. Egyptian physical therapists showed a very good knowledge about COVID-19. Most of them were aware that COVID-19 spreads by droplets of the affected person (with cough or expiration) and by surfaces touched by the affected person. Additionally, most of them had an awareness of the common symptoms of COVID-19 including fever, dry cough, and difficulty in breathing. Moreover, most of them had sufficient awareness of the measures that prevent the spread of COVID-19 such as proper hand washing, maintaining an appropriate physical distancing with symptomatic patients, and avoiding touching eyes, nose, and mouth. The mean total knowledge score was 18.29 out of 23, which is higher than the score of the public Egyptian population (16.39) [13]. The good knowledge about COVID-19 among Egyptian physical therapists presented in our study is consistent with previous studies conducted on Saudi physical therapists [18] and Egyptian healthcare workers [14].

Strengths and limitations

Our study is the first to investigate the impact of COVID-19 on clinical practices among physical therapists in Egypt, which adds important information to the literature. The study included a substantial number of participants (409 physical therapists) from 23 out of 27 Egyptian governorates. This broad geographic coverage enhances the generalizability of the findings within the country. However, convenient sampling may not accurately represent the population and may lead to selection bias. Moreover, as a cross-sectional study, it provides a snapshot of the situation at a specific point in time (August to October 2020). It does not account for changes over time or capture the long-term impact of the pandemic on physical therapy practice.

Recommendations

Physical therapists should be aware of precautionary measures against infectious diseases, which can help prevent the spread of disease if any new pandemic occurs.

## Conclusions

The COVID-19 pandemic affected physical therapy clinical practice in Egypt and had a psychological impact on Egyptian physical therapists. Egyptian physical therapists committed to precautionary measures against COVID-19 and demonstrated a very good knowledge about COVID-19. Physical therapists should be aware of precautionary measures against infectious diseases, which help prevent the spread of disease if any new pandemic occurs.

## Appendices

**Table 5:** Questionnaire on the impact of the COVID-19 pandemic on physical therapy clinical practice

Section 1: Demographic characteristics		
	Correct answer	
What is your gender?		
Male		
Female		
What is your age?		
What is your governorate of work?		
What is your area of work?		
Urban		
Rural		
What is your level of education? (Only one answer is allowed)		
Intern		
Bachelor's degree		
Doctor of physical therapy (DPT)		
Master of science (MSc)		
Doctor of philosophy (PhD)		
How many years of experience do you have?		
What is your scope of practice? (Multiple answers are allowed)		
Orthopedics		
Neurology		
Pediatrics		
Sports		
Geriatrics		
Cardiovascular and pulmonary		
Women's health		
Wound management		
Others, add		
What is your workplace? (Multiple answers are allowed)		
Ministry of Health and Population hospitals		
University hospitals		
Private centers		
Others		
Section 2: Interaction of physical therapists during the COVID-19 pandemic		
	Yes	No
Did you leave your work as a physical therapist at any period during the COVID-19 pandemic?		
Do you visit your patient's home "home physiotherapy," if requested?		
Are you afraid to catch any infection from patients during assessment and treatment?		
Do you feel anxiety about COVID-19 pandemic?		
Do you feel that your mental health and well-being are not okay?		
Section 3: What are the precautionary measures that you committed during assessment and treatment sessions?		
	Yes	No
Committing patients to wear face masks		
Committing patients to sterilize their hands before assessment and treatment		
Screening patient temperature		
Wearing face mask		
Wearing hand gloves		
Washing hands before and after every patient		
Cleaning and sterilizing assessment and treatment area including plinths, tools, and equipment before and after every patient		
Modifying techniques to keep social distance		
Section 4: Knowledge of physical therapists about COVID-19		
	Yes	No
COVID-19 spreads by		
1. Droplets of an affected person (with cough or expiration)		
2. Surfaces touched by an affected person		
3. Touching coins and banknotes		
4. Dealing with pets		
5. Stool (e.g., in public toilets)		
6. Goods imported from China		
7. The disease could be transmitted from an asymptomatic person		
Common symptoms include		
8. Fever		
9. Dry cough		
10. Body aches		
11. Difficulty in breathing		
12. Vomiting		
13. The virus may be more dangerous for the elderly		
14. The virus may be more dangerous in patients with chronic diseases		
Measures to prevent the spread of the disease include		
15. Proper hand wash		
16. Maintaining an appropriate distance between yourself and anyone with symptoms		
17. Avoiding touching eyes, nose, and mouth		
18. Putting on facemasks in public places		
19. Taking antibiotics		
20. Eating garlic		
21. An effective vaccine against the virus is currently available		
22. An effective treatment against the virus is currently available		
23. Antibiotics can treat the disease		
